The article "Security and Privacy Risk Assessment of Energy Big Data in Cloud Environment" was retracted in 2023. Reasons: signs of a paper mill; suspected computer-generated content; unreliable results or conclusions; concerns about the data.

# Security and Privacy Risk Assessment of Energy Big Data in Cloud Environment

**DOI:** 10.1155/2021/2398460

**Published:** 2021-10-14

**Authors:** Zhiru Li, Wei Xu, Huibin Shi, Yuanyuan Zhang, Yan Yan

**Affiliations:** ^1^Shenyang University of Technology, Shenyang, China; ^2^Dalian Medical University, Dalian, China

## Abstract

Considering the importance of energy in our lives and its impact on other critical infrastructures, this paper starts from the whole life cycle of big data and divides the security and privacy risk factors of energy big data into five stages: data collection, data transmission, data storage, data use, and data destruction. Integrating into the consideration of cloud environment, this paper fully analyzes the risk factors of each stage and establishes a risk assessment index system for the security and privacy of energy big data. According to the different degrees of risk impact, AHP method is used to give indexes weights, genetic algorithm is used to optimize the initial weights and thresholds of BP neural network, and then the optimized weights and thresholds are given to BP neural network, and the evaluation samples in the database are used to train it. Then, the trained model is used to evaluate a case to verify the applicability of the model.

## 1. Introduction

In the era of big data, the application of big data technology in the energy field is a trend to promote industrial development and innovation. Both the deep application of big data technology in the energy field and the deep integration of energy production, consumption, and related technology revolution with big data concept will accelerate the development of energy industry [1].

With the implementation of the global energy big data strategy, the rapid development of “Internet plus” smart energy and the comprehensive construction of intelligent energy layout make the energy industry more widely distributed, more data collection points, more data types, more complex business relationships, and a wider range of data usage and users [2]. So while bringing convenience, it also brings risks to energy big data management. Due to the critical infrastructure of each country, energy is bound to become the preferred target of attack in case of cyber war. With the frequent occurrence of more and more energy security and privacy incidents, such as “Blackout in Ukraine” and “Stuxnet virus” attack on Iran's nuclear facilities, big data has become a usable and attachable carrier [3]. Through the big data value information obtained by the attack, the energy distribution of the target location can be analyzed, and the key data such as the monitoring and early warning information and operation instructions of key nodes will be tampered, resulting in energy system failure or major security accidents.

Therefore, the management research based on energy big data has been widely concerned by scholars all over the world. At present, for the huge amount of data and the particularity of management in the energy industry, scholars carry out data management and architecture design through various technical or nontechnical means, including the establishment of big data layer to store and process renewable energy data [4] and the establishment of energy big data processing system, supporting memory distributed computing [5]. In the research on the security and privacy of big data, it is found that most scholars used a single model for risk assessment, such as analytic hierarchy process (AHP), factor analysis, grey theory [6], fuzzy evaluation method [7], and cloud model [8]. Such methods are based on statistical theory and cannot completely get rid of the influence of subjectivity and theoretical assumptions. In recent years, machine learning has become an important research tool in the field of security and privacy [9]. When using machine learning methods to evaluate and predict risks, the accuracy is often higher than that of traditional statistical methods [10]. Common machine learning methods include neural network, SVM, and clustering algorithm; BP neural network is the most widely used neural network in risk prediction and evaluation [11], but which is easy to fall into local minimum in practical application [12]. Therefore, scholars often use other algorithms as assistance to improve the accuracy of prediction and evaluation. For example, Zhang (2021) established a regression model through BP network and used PSO algorithm to optimize connection weights to evaluate the slow convergence of BP network, in order to improve the accuracy of rockburst prediction [13]. Wang (2019) et al. used LM algorithm to improve the operation efficiency and accuracy of traditional BP neural network and provided an effective theoretical basis and modeling method for risk prediction of power communication network [14].

This greatly improves the accuracy of prediction and evaluation, but a review of the relevant literature shows that the analysis of the importance of the impact of indexes is often neglected. Thus, in this paper, based on the consideration of machine learning, according to the different degrees of risk impact, AHP method is used to determine the index weight, which overcomes the deficiency of subjective consideration in previous studies [15]; the genetic algorithm optimized BP neural network (hereinafter referred to as GABP) with better prediction and evaluation effect is used for evaluation [16], which is a successful attempt to realize the combination of energy field and deep learning. In addition, for the security and privacy risk assessment of energy big data, the current literature pays more attention to theoretical analysis and lacks a relatively perfect assessment reference system. Starting from the whole life cycle of big data and considering the cloud environment, this paper establishes a risk assessment index system of energy big data security and privacy, which enriches the theoretical basis and framework in this field to a certain extent.

## 2. The Index System of Security and Privacy Risk Assessment of Energy Big Data in Cloud Environment

### 2.1. Principles for the Construction of the Index System

In the process of risk assessment, the probability of risk occurrence, loss range, and other factors need to be considered comprehensively to get the possibility and degree of system risk occurrence, determine the risk level, and then decide whether to take corresponding control measures and to what extent [17].

Therefore, the construction of risk assessment index system should follow the principles of comprehensiveness, scientificity, representativeness, and practicability, select the representative risk elements from a scientific perspective, quantify the risk based on the practical principle, and strive to show the risk management level comprehensively and accurately.

### 2.2. Identification of Risk Factors

Data security management is the most prominent risk faced by big data application. Although the massive data is stored centrally, it is convenient for data analysis and processing, but the loss and damage of big data caused by improper security management will cause devastating disaster. Due to the development of new technology and new business, the infringement of privacy right is not limited to physical and compulsory invasion, but is derived in a subtler way through various data, and the data security and privacy risks caused by this will be more serious [18].

Compared with the previous Internet and computer technology, the application advantage of big data in the cloud environment is more obvious. Big data platform has strong sharing ability, which can manage the security of information use and improve the efficiency of resource utilization. The construction of cloud platform and system application have strict standards. Cloud computing technology provides more comprehensive technical support and makes privacy management more reasonable, which is consistent with the level of technology development in the new era [19]. But from another point of view, it is under the influence of cloud platform sharing features that part of the data information is easy to be exposed, which provides opportunities for some illegal intrusion. Therefore, we must pay full attention to its risks.

Based on the literature of Xu [20], Tawalbeh [21], and He [22], combined with the analysis of relevant cases and the consultation of professionals, this paper follows the above evaluation index setting principle, combines with the development characteristics of energy big data security factors, and considers the impact of cloud environment. From the perspective of the whole life cycle of big data, this paper summarizes the current privacy security risks of cloud computing and big data and divides the risk assessment factors into five stages: data collection, data transmission, data storage, data use, and data destruction, with a total of 22 indexes, as shown in Figure 1.

### 2.3. Index Quantification

In terms of data collection, for the quantification of energy big data security and privacy risk indexes, this study introduces the concept of risk degree. According to the occurrence possibility and loss degree of each risk index, the product of possibility and loss degree is used as the reference standard of risk degree quantification, and the specific value can be reasonably floating around the product. The quantification of probability and loss degree can be divided into five levels: very high risk (5 points), high risk (4 points), medium risk (3 points), low risk (2 points), and very low risk (1 point).

(1) $$\begin{array}{c} R=P*L. \end{array}$$

In formula (1), *P* is the probability of occurrence and *L* is the degree of loss.

The normalized input value is multiplied by the corresponding weight of each index as the input of the neural network for training, combined with the output value; the risk assessment level can be obtained, as shown in Table 1.

## 3. Assessment Model of Energy Big Data Security and Privacy Risk in Cloud Environment

### 3.1. AHP Method

In the existing BP neural network part of the process, all kinds of risk factors are default to the same degree of impact, without a rigorous distinction, which is adverse to the establishment of neural network model.

Considering the particularity of energy big data security and privacy risk, quantitative analysis method may not be able to reasonably determine the real impact degree of indexes. Therefore, AHP method is used to give weight to indexes in this paper, and various factors in complex problems are divided into interconnected and ordered levels to make them methodical. According to the subjective judgment structure of certain objective reality, the expert opinions and the objective judgment results of analysts are directly and effectively combined, and the importance of pairwise comparison of one level elements is quantitatively described.

Therefore, after the establishment of energy big data security privacy and risk assessment index system, according to the influence degree of each risk factors, the Delphi method is used to invite experts to quantify the importance between them, and the AHP method is used to give corresponding weights to 22 indexes.

(1) Construct the judgment matrix.
The judgment matrix *A* = (*a*_*ij*_)*n∗n* is established by pairwise comparison. In order to make the judgment quantitative, the quantitative scale is given for the evaluation of different situations. The scale specification is shown in Table 2.
(2) Calculate the eigenvalue and eigenvector by the square root method and calculate the product of elements in each row of judgment matrix.
  (2) $$\begin{array}{c} M_{i}=\prod_{j=1}^{n}a_{ij}\left(i=1,2,\ldots ,n\right). \end{array}$$
Calculate the *n*th root of *M*_*i*_.
  (3) $$\begin{array}{c} \bar{W_{i}}=\sqrt[{n}]{M_{i}}\left(i=1,2,\ldots ,n\right). \end{array}$$
Normalize the eigenvectors as the weight.
  (4) $$\begin{array}{c} W_{A}={\left[W_{1},W_{2},\ldots ,W_{n}\right]}^{T}. \end{array}$$
Calculate the largest eigenvalue, where (AW)_*i*_ is the *i*th component of the vector AW.
  (5) $$\begin{array}{c} \lambda_{\max}=\overset{n}{\underset{i=1}{\sum }}\frac{{\left(\text{AW}\right)}_{i}}{nW_{i}}. \end{array}$$
(3) Check for consistency.

The consistency index *C.I.* is

(6) $$\begin{array}{c} C.I.=\frac{\lambda_{\max}-n}{n-1}. \end{array}$$

Generally, *C*.*I*.≤0.10 represents that the judgment matrix is consistent.

Obviously, with the increase of value *n*, the judgment error will increase, so the influence of *n* should be considered when judging the consistency, and the random consistency ratio *C*.*R*.=*C*.*I*./*R*.*I*. should be used, where *R.I.* is the average random consistency index.  Table 3 shows the average random consistency index test values calculated by the judgment matrix.

### 3.2. BP Neural Network

BP neural network is a kind of multilayer neural network, which was proposed by Rumelhart in 1986. It is one of the most widely used neural network models at present. It can learn and store a large number of input-output pattern mapping relations. Its learning rule is to use the steepest descent method to continuously adjust the weights and thresholds of the network through back propagation, so as to minimize the mean squared errors of the network. It is usually composed of input layer, hidden layer, and output layer [23], and its network model is shown in Figure 2.

The basic unit of neural network is neuron. The principle formula is shown in formula (7); the commonly used activation functions are threshold function, sigmoid function, and hyperbolic tangent function. In formula (7), the input of neurons is represented by *x*_*i*_ (*i* = 1, 2,…, *n*), the connection weights between neurons are represented by *w*_*i*_ (*i* = 1, 2,…, *n*), the threshold of neurons is *b*, the activation function is *f*, and the output of neurons is *y*.

(7) $$\begin{array}{c} y=f\left(\sum_{i=1}^{n}x_{i}w_{i}+b\right). \end{array}$$

For BP neural network, the mean square error *E* is often used as the index to judge the training performance of the model, shown in formula (8). The principle of minimizing the mean square error by adjusting the network weights is shown in formula (9), where *e* is the network error vector, *y*_*i*_ is the model output, and *t*_*i*_ is the target output.

(8) $$\begin{array}{c} E=\frac{1}{n}\sum_{i=1}^{n}w_{i}{\left(y_{i}-{\hat{y}}_{i}\right)}^{2}. \end{array}$$

(9) $$\begin{array}{c} \min E\left(e^{T}e\right)=\min E\left[{\left(t-y\right)}^{T}\left(t-y\right)\right]. \end{array}$$

For the training model, the LM algorithm of neural network is used in this study. The basic method to reduce the error is as follows:

(10) $$\begin{array}{c} x\left(k+1\right)=x\left(k\right)-{\left(J^{T}J+\mu J\right)}^{-1}J^{T}e,\\ J^{T}J=H, \end{array}$$

where *H* is the Jacobi matrix of the first derivative of the MSE function with respect to weights and thresholds.

### 3.3. Genetic Algorithm

Genetic algorithm (GA) is a computational model simulating the natural selection and genetic mechanism of Darwinian biological evolution theory. It is a method to search the optimal solution by simulating the natural evolution process [24].

Using genetic algorithm to get the optimal network weights and thresholds as the initial network weights and thresholds of the subsequent neural network model can not only overcome the defect that the traditional BP neural network is easy to fall into the local minimum, but also greatly improve the accuracy of model evaluation, so that the optimized BP neural network can better evaluate the samples. The elements of genetic algorithm include population initialization, fitness function, selection operator, crossover operator, and mutation operator.

Compared with binary coding, real coding can significantly reduce the length of coding and avoid the later decoding, with high accuracy. A series of parameters to be optimized, such as the connection weight, hidden layer node threshold, and output layer node threshold, are encoded by the s-order real matrix with the value range of [−1, 1].

After coding, the selection, crossover, and mutation are performed. These three operations are based on the fitness value calculated by the fitness function as the assessment standard. The smaller the value, the larger the fitness value, and the better the individual. The fitness function of this study is the reciprocal of mean square error function, as follows:

(11) $$\begin{array}{c} F\left[f\left(x\right)\right]=\frac{1}{f\left(x\right)}. \end{array}$$

In the selection operation, the most common roulette method is used. The probability of each individual being selected is positively proportional to its fitness value. *N* represents the population size, *F*_*i*_ represents the fitness function value of individual *i*, and *p*_*i*_ represents the probability of the *i*th individual being selected. The calculation way is as follows:

(12) $$\begin{array}{c} p_{i}=\frac{F_{i}}{\sum_{j=1}^{N}F_{j}}. \end{array}$$

By using arithmetic crossover as formula (13), a new individual is obtained by using the linear combination between two individuals, where *d* is a random number uniformly distributed in [0, 1]:

(13) $$\begin{array}{c} c_{1}=p_{1}*d+p_{2}*\left(1-d\right),\\ c_{2}=p_{1}*\left(1-d\right)+p_{2}*d. \end{array}$$

Mutation operation refers to the random mutation of individual gene of the population, enhancing the local search ability of the algorithm and maintaining the diversity of individual population. The operation method of mutation of the *j* gene of the *i* individual *a*_*ij*_ is as follows:

(14) $$\begin{array}{c} a_{ij}=\left\{\begin{array}{cc} a_{ij}+\left(a_{ij}-a_{\max}\right)*f\left(g\right), & r\geq 0.5,\\ a_{ij}+\left(a_{\min}-a_{ij}\right)*f\left(g\right), & r<0.5, \end{array}\right. \end{array}$$

where *a*_max_ is the upper bound of gene *a*_*ij*_, *a*_min_ is the lower bound of gene *a*_*ij*_*f*(*g*)=*r*_2_(1 − *g*/*G*_max_)^2^, *r*_2_ is a random number, *g* is the current iteration number, *G*_max_ is the maximum evolution number, and *r* is the random number of [0, 1] interval.

### 3.4. Construction of AHP-GABP Model

Compared with the traditional BP neural network, GABP model has a process of using genetic algorithm to optimize the weights and thresholds of the network, and this process can optimize the prediction performance of BP neural network to a certain extent. At the same time, using the AHP method to confirm the indicator weights can better define the importance of indicators. The flowchart is shown in Figure 3. The steps to build the AHP-GABP model are as follows:

1. Use AHP method to process data.
2. Determine the topological structure of BP neural network.
3. After the weights are given by AHP, determine the input and output sample set and test sample set of training.
4. The network parameters to be optimized are real-coded to form their own chromosomes.
5. Determine the parameters of selection, crossover, and mutation.
6. Set the population size popu.
7. After inputting samples, each chromosome produces corresponding output after network transmission.
8. The fitness value of each chromosome is calculated by fitness function, and the selection operation is carried out according to the fitness value.
9. A new generation of population is generated by crossover and mutation.
10. Repeat steps 6–8 until the fitness value of the optimal individual and the fitness value of the population do not rise within the specified number interval, or the fitness value of the optimal individual reaches the set threshold, or the number of iterations reaches the algebra set in advance, the algorithm stops, and the optimized network parameters are obtained.

## 4. Evaluation Process

### 4.1. Model Training

#### 4.1.1. Network Design

*(1) Network Structure Determination*. The paper selects 22 assessment indexes to assess the security and privacy risk of energy big data, so the number of input layer nodes is 22. In general, if the number of hidden layers is more, the error of assessment results will be smaller, but it will also bring the disadvantages of network complexity, thus reducing the efficiency of training [25]. For the multi-input single-output network model established in this paper, in order to increase the approximation effect and convergence, and reduce the oscillation in the simulation process, the number of hidden layer nodes is determined by referring to equation (15) and combining with the actual simulation results.

(15) $$\begin{array}{c} S_{1}=\sqrt{m+n}+a, \end{array}$$

where *m* represents the number of input layer nodes, *n* represents the number of output layer nodes, *a* takes a random integer between 1 and 10, and *S*_1_ = 12 is determined after trial calculation. The final MATLAB structure is shown in Figure 4.

*(2) Parameter Setting*. This study uses feedforward net to create function, trainlm to train function, logsig to transfer function, sigmoid to activate function, and MSE to express error *E.* The training times is 100, the learning rate is 0.01, and the training error target is 0.01. For the part of genetic algorithm, the number of population is set to 100, the maximum evolution algebra is set to 100, the variable precision is 1*e* − 6, the crossover probability is 0.8, and the mutation probability is 0.2.

#### 4.1.2. Training Results

After reading the literature and cases about the security and privacy risk of energy big data, a total of 44 samples are collected, including 36 training samples and 8 test samples. Some of the training data are shown in Table 4. The model training is realized by MATLAB programming and the development of Goat genetic algorithm toolbox.

The training data is input into the program, and the convergence curve of genetic algorithm optimized BP neural network is shown in Figure 5. It can be seen from the figure that the BP neural network algorithm after genetic algorithm optimization finds an optimal path optimal solution when the population iteration is about 60 generations, which shows the superiority of genetic algorithm in optimizing the weight and threshold of BP neural network. It can also be seen that the optimal function tends to be stable when the iteration reaches nearly 70 generations.

The BP neural network and the optimized genetic BP neural network are compared, and their error values are calculated. The final experimental results are shown in Table 5. Through analysis and comparison, in 8 groups of test samples, AHP-GABP prediction has significant advantages over BP prediction, with smaller error, shorter evaluation cycle, and greater improvement in evaluation performance. As shown in Table 5 and Figure 6, the BP neural network optimized by genetic algorithm improves the shortcomings of BP neural network, thus greatly improving the predictability of neural network. At the same time, the application assessment results of the BP neural network optimized by genetic algorithm in the energy big data security and privacy risk are basically consistent with the actual expert assessment results, which proves that the training network has high accuracy.

### 4.2. Model Applications

#### 4.2.1. Background

Z power grid system uses its energy big data information to provide data services related to economic development. It can provide more reliable data support for poverty alleviation effect evaluation, credit evaluation, census, pollution monitoring, and work resumption evaluation. According to the energy big data security and privacy risk assessment index system designed above, the complete evaluation steps of big data security and privacy risk of this power grid system are as follows:

- Calculate the index weights using AHP method.
- Collect relevant data of this grid system, invite relevant department heads to score the 22 risk assessment indicators, and standardize the data with the weights as the input values of the AHP-GABP model.
- Use the above trained AHP-GABP network model; the output values are evaluated, and the risk level is defined according to the risk classification method.

#### 4.2.2. Initial Index Weight of AHP Method

In this study, AHP method is used to assign weights to the primary and secondary indexes, respectively. After the consistency check, the final weights of 22 indexes are obtained as shown in Table 6.

#### 4.2.3. Assessment Results

In this study, three groups of relevant data collected by the power grid system are selected. After training, the AHP-GABP neural network model is established. Firstly, it is necessary to verify whether the evaluation model is reasonable. Secondly, it is necessary to assess the risk. The assessment results are shown in Table 7, which shows that the risk level of the power grid system is class 1, which is similar to the conventional risk performance of the power grid system. The risk level is low, and there is no need to do special treatment, and regular inspection should be done. It also shows that the AHP-GABP algorithm is reasonable and correct in the evaluation and prediction, with high prediction accuracy, objective and fair evaluation results, wide application range, and high practical application value.

## 5. Conclusion and Development Suggestions

To sum up, in the process of controlling the energy big data security and privacy risk, the risk of each stage cannot be ignored. On the premise of comprehensively considering the cloud environment and risk factors, this paper divides the potential energy big data security and privacy risk of each stage as comprehensively as possible according to the life cycle of big data, and uses AHP method to allocate weights for the indexes, which provides a reference for the future energy big data research. At the same time, this paper optimizes the BP neural network model based on the evaluation, and tries to apply the AHP-GABP method to the risk evaluation of energy big data security and privacy, which greatly reduces the risk that the random selection of initial weights and thresholds in BP algorithm leads to the model training easily falling into the local minimum, and improves the accuracy of neural network model assessment and predication and realizes the application of AI related knowledge in the field of energy.

The AHP-GABP model is applied to evaluate the security and privacy of the energy big data, and the evaluation results are good. According to the case and expert interviews, the following development suggestions are summarized for the common risks of energy big data security and privacy.

### 5.1. Pay Attention to the Security of the Whole Life Cycle of Energy Big Data

Energy big data comes from production data and operation and management data, and its protection should focus on the whole life cycle of data collection, transmission, storage, use, and destruction. From policy and system requirements to technical management and control, we should comprehensively assess the threat exposure of critical data and make targeted protection strategies at all stages to ensure the security of core data assets.

### 5.2. Strengthen Technical Protection of Energy Industry Based on Big Data Security

The energy industry should establish a comprehensive threat early warning technology based on security big data, break through the traditional mode, and more actively detect potential security threats. The introduction of big data analysis technology in threat detection can more comprehensively detect attacks on data assets, software assets, physical assets, personnel assets, service assets, and other intangible assets supporting business [26]. At the same time, the scope of the analysis content can be expanded. The threat analysis window can span several years of data, so the threat detection ability is stronger and can effectively respond to the attack [27].

### 5.3. Consider Security and Privacy Issues from a Strategic and Long-Term Perspective

Big data brings opportunities and challenges to the energy industry. The more widely it is applied, the greater the value it brings. The concept of security management centered on data security will change the traditional working ideas [28]. We must recognize the new changes, new features, and new trends of big data security, and deeply analyze the outstanding problems existing in big data security under the current situation. In order to ensure that the development strategy of energy big data information security is consistent with the national conditions and constantly improves, it is necessary to plan the key layout of big data application, key technology research and development, data protection, laws and regulations.

With the rapid development of cloud computing and the continuous improvement of digital level, the energy big data security and privacy risk evaluation index system can be further improved. At the same time, with the enrichment of data indicators and training models, the model proposed in this paper can also be better optimized and expanded to other fields for more accurate evaluation and prediction in the future.

## Figures and Tables

**Figure 1:** Security and privacy risk assessment index system based on the whole life cycle of energy big data.

**Figure 2:** Structural model of neural network.

**Figure 3:** AHP-GABP flowchart.

**Figure 4:** MATLAB structure.

**Figure 5:** Fitness value.

**Figure 6:** Error comparison between predictive value and real value.

**Table 1:** Risk assessment level.

Risk level	Meaning
First class (0 ≤ *R ≤* 0.2)	The risk level is very low, so it is not necessary to pay special attention to it. The plan and general prevention can be made.
Second class (0.2 < *R* ≤ 0.4)	The risk level is low, the plan and general prevention should be made, and need to be checked regularly.
Third class (0.4 < *R* ≤ 0.6)	The risk level is medium; the major risk factors should be paid attention to in combination with the specific situation, and the corresponding countermeasures should be formulated.
Fourth class (0.6 < *R* ≤ 0.8)	The risk level is high; it is necessary to pay attention to all the risk factors that may threaten the security of energy data, formulate the process sequence after the occurrence of the risk according to the importance degree, and track the inspection and evaluation.
Fifth class (0.8 < *R* ≤ 1.0)	The risk level is very high; if necessary, it can be stopped and maintained, and the comprehensive inspection and special evaluation should be carried out immediately and can be continued after improvement.

**Table 2:** Scale specification.

Scale	Meaning (*a*_*i*_ vs *a*_*j*_)
1	The former is as important as the latter
3	The former is slightly more important than the latter
5	The former is obviously more important than the latter
7	The former is strongly more important than the latter
9	The former extremely is more important than the latter
2, 4, 6, and 8	The intermediate value of the above two adjacent judgments
The reciprocal of the above values	If the ratio of factors *i* and *j* is *a*_*ij*_, then the factor of the ratio of factors *j* and *i* is *a*_*ji*_ = 1/*a*_*ij*_

**Table 3:** *R.I.* value.

Order number	1	2	3	4	5	6	7	8	9	10
*R.I.*	0	0	0.58	0.90	1.12	1.24	1.32	1.41	1.45	1.49

**Table 4:** Training samples.

	1	2	3	4	5	6	7	8
A1	0.7028	0.5020	0.6024	0.6526	0.5522	0.6024	0.6024	0.5522
A2	0.3784	0.8514	0.9933	1.0406	0.6622	0.6622	0.6149	0.2838
A3	0.5400	0.2700	0.7200	0.8100	0.4050	0.2700	0.4500	0.1800
A4	0.3612	0.3010	0.4515	0.5418	0.2408	0.3010	0.3311	0.2408
B1	0.0516	0.0344	0.1290	0.1290	0.0688	0.0774	0.0688	0.0430
B2	0.0748	0.0408	0.1088	0.1360	0.0680	0.0816	0.0476	0.0476
B3	1.4922	0.9948	1.9067	0.9948	1.4922	1.2435	1.0777	0.9948
B4	1.9100	2.1965	2.0055	1.1460	2.0055	1.2415	1.3370	0.9550
B5	0.4992	0.6240	0.5408	0.3328	0.5824	0.2496	0.4160	0.2496
C1	0.1854	0.4326	0.4326	0.1545	0.5871	0.3090	0.2781	0.2163
C2	0.0648	0.1620	0.1944	0.0810	0.2430	0.1134	0.1134	0.0486
C3	1.6300	1.6300	2.2820	1.6300	1.9560	1.7930	1.6300	1.4670
C4	1.8032	1.0304	2.0608	0.7728	1.2880	2.7048	1.8032	1.2880
C5	0.5130	0.5130	1.0260	0.4617	0.5130	0.9747	0.4104	0.4104
D1	0.2808	0.5967	0.6318	0.2808	0.3159	0.5265	0.2106	0.3159
D2	0.5136	0.3531	0.6741	0.3210	0.3210	0.6420	0.2247	0.2247
D3	0.1932	0.1380	0.2208	0.0966	0.0828	0.2346	0.0966	0.0828
D4	0.3108	0.4144	0.3626	0.2331	0.1813	0.4662	0.2072	0.2072
D5	0.2100	0.2520	0.1680	0.1260	0.1680	0.3360	0.1260	0.1680
E1	0.7434	0.2891	0.7847	0.4956	0.4130	0.5369	0.8260	0.4130
E2	0.1261	0.1164	0.1358	0.0970	0.0582	0.1358	0.1552	0.0582
E3	0.0156	0.0117	0.0312	0.0156	0.0195	0.0234	0.0546	0.0234
Output	0.7813	0.7558	0.9149	0.6012	0.7801	0.7889	0.5989	0.4569
Risk level	4	4	5	4	4	4	3	3

**Table 5:** Comparison of training sample error between BP neural network and AHP-GABP neural network.

Sample number	Real value	Predictive value		Error	
		BP	AHP-GABP	BP	AHP-GABP
1	0.7813	1.4328	0.7717	0.6515	−0.0096
2	0.7558	0.4292	0.7443	−0.3266	−0.0115
3	0.9149	1.9229	0.8984	1.0080	−0.0165
4	0.6012	−1.0077	0.5324	−1.6089	−0.0688
5	0.7801	0.3213	0.7503	−0.4588	−0.0298
6	0.7889	0.7989	0.8125	0.0100	0.0236
7	0.5989	1.3607	0.5810	0.7618	−0.0179
8	0.4569	−0.0912	0.4442	−0.5481	−0.0127

**Table 6:** Weights of risk assessment indexes.

First-level index	Second-level index	Weight
Data collection A	Software and hardware fault risk A1	0.0601
	Damage or consumption risk of energy infrastructure A2	0.0270
	External malicious attack A3	0.1058
	Irresistible force risk A4	0.0108

Data transmission B	Malicious intercepting risk B1	0.1774
	Malicious tampering risk B2	0.1133
	Data distortion risk B3	0.0720
	Access control risk B4	0.0210
	Cloud platform risk B5	0.0317

Data storage C	Sleeping data risk C1	0.0124
	Quality of data input risk C2	0.0163
	Data leakage risk C3	0.1237
	Management data destruction risk C4	0.0324
	Virus intrusion risk C5	0.0680

Data use D	Multi source data fusion risk D1	0.0432
	Privacy awareness of business personnel D2	0.0046
	Data parsing risk D3	0.0113
	Data regulatory risk D4	0.0165
	Manage authorization risk D5	0.0071

Data destruction E	Data residual risk E1	0.0135
	Data backup risk E2	0.0245
	Termination of cloud service agreement risk E3	0.0074

**Table 7:** Case assessment result.

Sample	AHP-GABP result	Risk level
1	0.1710	1
2	0.1715	1
3	0.1033	1

## Data Availability

The data used to support the findings of this study are available from the corresponding author upon request.

## References

[1] Ouadine A. Y., Mjahed M., Ayad H., El Kari A. (2020). UAV quadrotor fault detection and isolation using artificial neural network and hammerstein-wiener model. *Studies in Informatics and Control*.

[2] Fu L., Dong Y. (2018). Research on internet search data in China’s social problems under the background of big data. *Journal of Logistics, Informatics and Service Science*.

[3] Banciu D., Rădoi M., Belloiu S. (2020). Information security awareness in Romanian public administration: an exploratory case study. *Studies in Informatics and Control*.

[4] Naoui M. A., Brahim L., Ayad M. (2020). Integrating iot devices and deep learning for renewable energy in big data system. *UPB Scientific Bulletin, Series C: Electrical Times*.

[5] Song M. (2018). Development of big data system for energy big data. *KIISE Transactions on Computing Practices*.

[6] Mendonça Silva M., Poleto T., Camara e Silva L., Henriques de Gusmao A. P., Cabral Seixas Costa A. P. (2016). A grey theory based approach to big data risk management using fmea. *Mathematical Problems in Engineering*.

[7] Fu Y., Wu X. . p., Ye Q., Peng X. (2010). An approach for information systems security risk assessment on fuzzy set and entropy-weight. *Acta Electronica Sinica*.

[8] Chen L., Pan H.-Y. (2013). Cloud-model based decision-making for network risk assessment. *Journal of Computer Applications*.

[9] Sagar R., Jhaveri R., Borrego C. (2020). Applications in security and evasions in machine learning: a survey. *Electronics*.

[10] Kim J. B. (2019). Implementation of artificial intelligence system and traditional system: a comparative study. *Journal of System and Management Sciences*.

[11] Öztürk A., Taşpinar F. (2019). Short term load forecasting for Turkey energy distribution system with artificial neural networks. *Tehnicki vjesnik - Technical Gazette*.

[12] Li S., Bi F., Chen W., Miao X., Liu J., Tang C. (2018). An improved information security risk assessments method for cyber-physical-social computing and networking. *IEEE Access*.

[13] Zhang M. (2021). Prediction of rockburst hazard based on particle swarm algorithm and neural network. *Neural Computing and Applications*.

[14] Wang Y., Wang K., Zhang R., Xue Q., Chen X., Zhang G. (2019). Risk assessment of power communication network based on LM-BP neural network. *Journal of Physics: Conference Series*.

[15] Wang L., Bi X. (2021). Risk assessment of knowledge fusion in an innovation ecosystem based on a ga-bp neural network. *Cognitive Systems Research*.

[16] Zhu C., Zhang J., Liu Y., Ma D., Li M., Xiang B. (2020). Comparison of GA-BP and PSO-BP neural network models with initial BP model for rainfall-induced landslides risk assessment in regional scale: a case study in Sichuan, China. *Natural Hazards*.

[17] Li Y., Xu M., Wen X., Guo D. (2020). The role of internet search index for tourist volume prediction based on gdfm model. *Tehnicki vjesnik - Technical Gazette*.

[18] Anthi E., Javed A., Rana O., Theodorakopoulos G. (2017). Secure data sharing and analysis in cloud-based energy management systems. *Cloud Infrastructures, Services, and IoT Systems for Smart Cities*.

[19] Bommala H., Kiran S. (2020). Cloud computing technology for digital economy. *i-manager’s Journal on Cloud Computing*.

[20] Lei Xu L., Chunxiao Jiang C., Jian Wang J., Jian Yuan J., Yong Ren Y. (2014). Information security in big data: privacy and data mining. *IEEE Access*.

[21] Tawalbeh L. a. A., Saldamli G. (2021). Reconsidering big data security and privacy in cloud and mobile cloud systems. *Journal of King Saud University - Computer and Information Sciences*.

[22] He Y., Ji J. (2021). Analysis of information security risk defense in the development of big data. *Journal of Physics: Conference Series*.

[23] Lorenc A., Kuźnar M., Lerher T., Szkoda M. (2020). Predicting the probability of cargo theft for individual cases in railway transport. *Tehnicki vjesnik - Technical Gazette*.

[24] Xing Y., Li F. (2020). Research on the influence of hidden layers on the prediction accuracy of GA-BP neural network. *Journal of Physics: Conference Series*.

[25] Qian Y. . s., Zeng J. . w., Zhang S. . f., Xu D. . j., Wei X. . t. (2020). Short-term traffic prediction based on genetic algorithm improved neural network. *Tehnicki vjesnik - Technical Gazette*.

[26] Tabsh Y., Davidavičien˙e V. (2019). Ict in energy security and efficiency assurance. *Journal of System and Management Sciences*.

[27] Fu Y., Li H., Wu X., Wang J. (2015). Detecting apt attacks: a survey from the perspective of big data analysis. *Journal on Communications*.

[28] Tijani N., Popoola O. D. (2019). Challenges and opportunities in organizational operations and research methods. *Journal of Logistics, Informatics and Service Science*.

